# Application of Microspectral Imaging in Motor and Sensory Nerve Classification

This article has been retracted.

**DOI:** 10.1155/2021/4954540

**Published:** 2021-12-06

**Authors:** Du Xu

**Affiliations:** Xi'an University of Posts and Telecommunications, Shanxi, Xi'an 710100, China

## Abstract

**Objective:**

It aimed to explore the application of the microscopic hyperspectral technique in motor and sensory nerve classification.

**Methods:**

The self-developed microscopic hyperspectral acquisition system was applied to collect the data of anterior and posterior spinal cord sections of white rabbits. The joint correction algorithm was employed to preprocess the collected data, such as noise reduction. On the basis of pure linear light source index, a new pixel purification algorithm based on cross contrast was proposed to extract more regions of interest, which was used for feature extraction of motor and sensory nerves. Besides, the ML algorithm was employed to classify motor and sensory nerves based on feature extraction results.

**Results:**

The joint correction algorithm was adopted to preprocess the data collected by the microscopic hyperspectral technique, so as to eliminate the influence of the incident light source and the system and improve the classification accuracy. The axon and myelin spectrum curves of the two kinds of nerves in the stained specimens had the same trend, but the values of all kinds of spectrum of sensory nerves were higher than those of motor nerves. However, the myelin sheath spectrum curves of motor nerves in the unstained specimens were greatly different from the curves of sensory nerves. The axon spectrum curves had the same trend, but the axon spectrum values of sensory nerves were higher than those of motor nerves. The ML algorithm had high accuracy and fast speed in motor and sensory nerve classification, and the classification effect of stained specimens was better than that of unstained specimens.

**Conclusion:**

The microscopic hyperspectral technique had high feasibility in sensory and motor nerve classification and was worthy of further research and promotion.

## 1. Introduction

Hyperspectral image data are defined as a narrow continuous spectrum obtained in the range of visible, near-infrared, mid-infrared, and far-infrared bands in the electromagnetic spectrum, which can be divided into spatial and spectral parts [1]. In recent years, the increasingly mature development of spectral imaging technology, coupled with its advantages of large amount of information and high resolution, has attracted more and more scholars to investigate its application in biomedical field [2]. At present, the research direction in this field mainly focuses on two aspects, namely, the imaging system based on the existing medical equipment and the data analysis research based on the collected data [3]. At present, the microscopic hyperspectral technique has been applied to the evaluation of the healing degree of injured skin, tumor localization and differentiation, melanoma diagnosis, and other aspects [4, 5].

Peripheral nerve injury mainly includes motor and sensory nerve injuries and is the most common cause of sensory and motor function loss in patients. The main treatment is to repair the damaged nerves. In order to ensure the repair effect of the injured nerve, the two broken nerves have to be accurately matched for mirror anastomosis [6]. What was more, the premise and basis of the implementation of this treatment is the accurate judgment of nerve type. At present, the frequently applied clinical methods for nerve bundle identification are the electrophysiological method, isotope method, anatomical method, and histological method. However, these methods have their own limitations, as they generally show the shortcoming of long detection time [7]. Therefore, a fast, efficient, accurate, specific, and simple neural recognition method is urgently needed. A large number of studies have shown that, theoretically speaking, microscopic hyperspectral technology has the advantages of simple operation, high accuracy, and fast detection speed in resolving neural velocity [8]. It indicates that the microscopic hyperspectral technique has great potential in differentiating nerve types, which has the value of further thorough and comprehensive research.

## 2. Research Methods and Materials

### 2.1. Research Objects

The spinal cord roots of white rabbits were frozen to make for sections. Moreover, the sections were divided into stained and unstained sections. All sections adopted in this study were provided by the Department of Orthopedics of X Hospital, which were made and processed by professional staff.

### 2.2. Collection of Microscopic Hyperspectral Image Data

The microscopic hyperspectral acquisition system used in this study was independently developed by xxx laboratory, which was composed of two parts (microscopy technique and spectroscopy technique). Spectral and microscopic information could be obtained simultaneously. Besides, the hardware was mainly formed with a microscope, acousto-optic tunable filter (AOTF) spectrometer, radio frequency (RF) driver, array charge coupled device (CCD) image acquisition card, and computer grade part. The software design of this system was based on C++ Builder 6.0, and the specific collection flowchart is shown in Figure 1. First step was that the magnification of the microscope was selected, and the intensity of the incident light source was adjusted as well as the position of the carrier section on the carrier stage, so as to make the target clearly visible in the eyepiece and the size appropriate. Second step was to judge whether it was the target object through the real-time display of the software platform. Third step was parameter setting, system initialization, selection of collection mode, and other operations. Fourth step was data collection.

### 2.3. Data Preprocessing

The differences of spectral data of biological tissue specimens were small, and the similarity between blank sections and tissue specimens was also great. This made the judgment more difficult, so it was necessary to reduce the interference factors and to preprocess the data such as noise reduction. In this study, the joint correction algorithm was adopted to process the data from two levels, that was, spectrum and space dimension.

The spectral dimension correction coefficient *k*_1_(*i*, *j*, *λ*) and spatial dimension correction coefficient *k*_2_ were obtained by using the original spectral data of blank section. Then, *k*_2_ and *k*_1_ were used and corrected the hyperspectral data of the white rabbit specimens. The size of the original blank hyperspectral was *M*•*N*•*L*. What was more, *M* and *N* represent the pixel values of hyperspectral data in two-dimensional space, and *L* represents the number of bands. In addition, *k*_1_(*i*, *j*, *λ*) could be expressed in the following equation.

(1) $$\begin{array}{c} k_{1}\left(i,j,\lambda \right)=\frac{\bar{B}\left(i,j\right)}{B\left(i,j,\lambda \right)}. \end{array}$$

*B*(*i*, *j*, *λ*) represents the light transmittance intensity value of the blank slide specimen at the point (*i*, *j*) on the band *λ*, and $\bar{B}\left(i,j\right)$ expresses the average value of the light transmittance intensity value of the blank specimen point (*i*, *j*) on all bands, which could be obtained from the following equation.

(2) $$\begin{array}{c} \bar{B}\left(i,j\right)=\frac{\sum_{\lambda =1}^{L}B\left(i,j,\lambda \right)}{L}. \end{array}$$

The expression of *k*_2_ is given in equation (3), $\bar{B}\left(i,j\right)$ could be calculated in equation (2), and *B* was the mean value of $\bar{B}\left(i,j\right)$. Thus, *B* is expressed in equation (4).

(3) $$\begin{array}{c} k_{2}=\frac{B}{\bar{B}\left(i,j\right)}, \end{array}$$

(4) $$\begin{array}{c} B=\frac{\sum_{j=1}^{N}\sum_{i=1}^{M}\bar{B}\left(i,j\right)}{M•N}. \end{array}$$

After joint correction, the original microscopic hyperspectral data *S*(*i*, *j*, *λ*) of white rabbits are expressed as

(5) $$\begin{array}{c} S^{\cdot }\left(i,j,\lambda \right)=S\left(i,j,\lambda \right)•k_{1}\left(i,j,\lambda \right)•k_{2}. \end{array}$$

### 2.4. Feature Extraction of Peripheral and Motor Nerve Specimen Data

The premise of feature extraction data analysis was the most critical step in the data analysis process. The extraction and analysis effect of all image information depended on the extracted feature information. The data extracted by the microscopic hyperspectral system were recorded in the form of pixels. A pixel could contain many forms because the microscope resolution or the specimen itself was a mixture of different types of nerves. It increased the difficulty of classification judgment. Therefore, it was necessary to purify pixels to obtain pure pixels for purification. First, the original hyperspectral data were dimensionalized to reduce noise and specimen size. The pixel purity index (PPI) was used for endmember mapping. Finally, the ultimate pure neurons of each type of nerve were extracted by N-dimensional visual analysis tools.

### 2.5. Classification of Motor and Sensory Nerves

According to the characteristics of motor and sensory nerve placement, the maximum likelihood algorithm was selected as the classification algorithm. The so-called maximum likelihood algorithm is a nonlinear algorithm that classifies the probabilities of the measured points to various categories. The maximum likelihood algorithm is suitable for the analysis of specimen data conforming to normal distribution. In line with the normal distribution random variable *X*, the probability density function can be expressed as

(6) $$\begin{array}{c} F\left(x\right)=\frac{1}{\sqrt{2\pi }\sigma }\int_{-\infty }^{x}e^{{\left(1-\mu \right)}^{2}/2\sigma^{2}}dt\left(-\infty <x<+\infty \right). \end{array}$$

The final discrimination algorithm of the maximum likelihood algorithm is shown in the following equation. Furthermore, *x* represents the input specimen. ∑_*i*_ and *μ*_*i*_ are the variance matrix and mean vector of the specimen set *D*_*i*_, respectively.

(7) $$\begin{array}{c} g_{i}\left(x\right)=InP\left(D_{i}\right)-In\left|\sum {}_{i}\right|-{\left(x-\mu_{i}\right)}^{T}\sum_{i}^{-1}\left(x-\mu_{i}\right)\;i=1...c. \end{array}$$

The classification decision function is presented in the following equation.

(8) $$\begin{array}{c} x\in D_{i}.fg_{i}\left(x\right)>g_{j}\left(x\right)\text{, for all }j\neq i. \end{array}$$

## 3. Results

### 3.1. Microscopic Hyperspectral Data Analysis

In this study, the collected microscopic hyperspectral data were analyzed from two aspects of spectrum and image dimensions. Through observation and analysis of the images collected from the white rabbit specimens and blank slides by the microscopic hyperspectral acquisition system, it was found that the images collected by the acquisition system had some trouble factors such as black spots, noise, and irregular stripes. It might be caused by dust in the optical path, which could be reduced by regular dust removal. Spectral data collected by the system are shown in Figures 2 and 3.

Figure 2 shows that the incident light intensity of the carrier slice with the specimen superposed at the same coordinate position was weaker than that of the blank slide.  Figure 3 shows that the spectral shapes of all kinds of tissues were manifested as the shape of incident light wave. This might be due to the thin and transparent nature of biological tissue. However, the attenuation degree of light wave was different in different coordinates of different biological tissues. Biological tissues could be classified by analyzing the attenuation of light waves. It was necessary to preprocess the collected data in order to achieve accurate and rapid classification.

### 3.2. Results of Image Preprocessing

The image performance of the neural specimens processed by the joint correction algorithm was the same as the original image, and the interference factors such as noise, gray spots, and bands were completely removed. After processing, the mean wave curves of the regions of interest are shown in Figure 4. It revealed that the background mean pop curve approximated a curve, and then, the mean pop curves of the regions of interest also had obvious differences. It was found that the joint correction algorithm had a good processing effect on the data collected by the microscopic hyperspectral technique.

### 3.3. Results of Pure Pixel Extraction

According to the above algorithm, pure pixel elements were extracted from the collected images, and then, the average value of various pure pixel elements was calculated to obtain their characteristic spectral curves, as shown in Figures 5 and 6. The motor and sensory axons, myelin sheaths, and background spectrum were very different, but the spectral curves of the two types of nerves showed the same pattern.

### 3.4. Effect Comparison of Maximum Likelihood Algorithm and Various Algorithms in Neural Classification

The comparison results of motor and sensory nerve classification and classification time among the maximum likelihood algorithm and other algorithms are given in Table 1. It indicated that × represents the poor classification effect and ↑ represents the classification effect level. The more the number, the better the classification effect. Table 1 provides that the maximum likelihood algorithm had the best classification accuracy in both stained and unstained specimens, with the advantage of fast classification speed.

## 4. Discussion

The application of spectral technology in biomedicine can be divided into two categories, including imaging diagnosis and spectral diagnosis. Both of these techniques can only obtain a single spectral and image result, thereby leading to single information, small quantity, and other shortcomings. By contrast, the microscopic spectral technique can obtain spectral and phase information simultaneously and has abundant information. In recent years, it has made great progress in the field of biomedical science due to the advantages of the microscopic spectral technique [9]. At present, a large number of scholars have investigated its application in the field of biomedical science. At present, the microscopic hyperspectral technique has been applied in clinical practice in dermatology diagnosis, tumor localization, and cell analysis [10–12].

At present, clinical methods for nerve classification mainly focus on electrophysiology and tissue characteristics [13]. There are few studies on the classification of old nerves using optical techniques. With the development of microscopic hyperspectral technology in the field of biomedical research, some scholars also proposed to apply it to neural classification. Some scholars employed the microscopic hyperspectral technique to collect images of the motor and sensory nerves of the anterior and posterior root sections of the spinal cord of dogs, so as to analyze the spectra. It was found that the spectral direction and trend of the two types of nerves were the same, but there was a big difference in the value of the spectrum curve [14]. This indicated that the microscopic hyperspectral technique had great potential and feasibility in the distinction between motor and sensory nerves.

In this study, a self-developed microscopic hyperspectral system was adopted to collect the data of the anterior and posterior roots of the spinal cord of white rabbits. Then, the images were preprocessed by the joint correction algorithm. Besides, the pure pixel was extracted from the data. Finally, motor and sensory nerves were classified by the maximum likelihood algorithm. Thus, a specific method of collecting motor and sensory nerves by the microscopic hyperspectral technique was proposed in this study. For the preprocessing and feature extraction of the collected images, the optimal scheme was given. In this study, an algorithm with high sensitivity, high classification speed, and high accuracy was presented for neural classification, and its feasibility needed to be studied. To a certain extent, the research on the application of the microscopic spectral technique in the motor and sensory nerve classification was enriched, so as to provide more possibilities for clinical nerve repair and diagnosis. It could be used as a supplement to the traditional neurodiagnostic methods. All the experiments in this study remain at the stage of specimen and are limited in length and specimen, so they are not comprehensive and in-depth. Further in-depth and comprehensive studies are needed if it is to be applied in clinical practice.

## 5. Conclusion

In this study, a self-developed microscopic hyperspectral system was applied to collect the data of the anterior and posterior roots of the spinal cord of white rabbits. Then, the images were preprocessed by the joint correction algorithm, and the pure pixel was extracted from the data. Finally, motor and sensory nerves were classified by the maximum likelihood algorithm. A method with high sensitivity, high classification speed, and high accuracy for motor and sensory nerve classification was presented in this study, and its feasibility was explored.

## Figures and Tables

**Figure 1:** Microscopic hyperspectral data acquisition process.

**Figure 2:** Spectral curves of blank slide and nerve specimens.

**Figure 3:** Spectral curves at different coordinates of nerve specimens.

**Figure 4:** Correction of neural mean pop curves with the joint algorithm.

**Figure 5:** The mean spectrum curves of motor nerves.

**Figure 6:** The mean spectrum curves of sensory nerves.

**Table 1:** Comparison on the neural classification effect among these algorithms.

Algorithm		Min. distance (S)	SVM (S)	ML (S)
Time		12.01	654.46	41.9
Classification performance	Stained specimens	↑	↑↑↑	↑↑↑
	Unstained specimens	×	↑	↑↑↑

## Data Availability

The data used to support the findings of this study are available from the corresponding author upon request.
